This article has been retracted.

# Pathological Clinical Analysis and Imaging Manifestations for Spinal Bone Tumors Based on Cement Injection

**DOI:** 10.1155/2022/2105332

**Published:** 2022-04-25

**Authors:** Jie Li, Xu Wang, Yongmin Li, Qinhui Cao, Yi Bu, Hengcong Cao, Xiaoqiang Wang

**Affiliations:** ^1^Department of Spine, Second Hospital of Tangshan, Tangshan, Hebei, China 063000; ^2^Department of Neurosurgery, Xinhua Hospital Affiliated to Shanghai Jiaotong University School of Medicine, Shanghai, China 200000

## Abstract

In order to explore the imaging manifestations and pathological characteristics of spine tumors, this article explores the clinical diagnosis and treatment methods through multi-sample case analysis with the support of imaging, and proposes a targeted treatment method that uses a special PVP needle with a beveled puncture surface for puncture. Moreover, this article uses the supporting PVP syringe for bone cement injection, develops a health status questionnaire, and adopts a scoring method for comprehensive assessment. The purpose of this article is to show that through the combination of preoperative radiotherapy and postoperative bracing, bone cement injection to treat vertebral tumors can immediately obtain satisfactory pain relief. Finally, through case analysis and image performance, we can see that the method proposed in this article has a certain effect.

## 1. Introduction

Bone metastases can occur in bones throughout the body, of which spinal metastases are the most common [1]. Patients with spinal metastases often suffer from severe pain, motor dysfunction, and even paralysis due to vertebral body destruction, pathological fractures, and tumor growth compressing the spinal cord and nerves. This seriously affects the patient's quality of life, reduces the patient's survival rate, and brings a heavy burden to the patient's family [2]. The treatment principle of vertebral metastasis is to relieve the pain of the patient, improve the patient's motor and nerve function, and improve the patient's quality of life. Single vertebral body metastasis can be treated by surgery, external radiotherapy, and other treatments. At present, the most commonly used treatment method for spinal metastases is external radiotherapy. The effective relief rate of external radiotherapy for pain caused by vertebral body destruction can reach 70%-90% [3]. If the lesion is close to the spinal cord, too much radiotherapy will damage the spinal cord and cause radiotherapy toxic reactions. If the dose is too small, it will not be effective in killing the tumor. Moreover, there is currently no uniform standard for radiotherapy methods and radiotherapy doses for bone metastases [4], and it is difficult to achieve decompression or stabilization with radiotherapy alone. There is a general consensus that surgery is recommended for patients with a survival expectancy of at least 3 months, and more than 24 hours of paraplegia is an exclusion criterion. Due to stricter selection criteria, surgery seems to be only suitable for 10% to 15% of patients. Moreover, surgery can easily cause complications including spinal cord or spinal root injury, extensive bleeding, infection, and dural tear. For multiple vertebral metastases, patients are often unable to withstand multi-site surgical operations, and there are few surgical indications, and most patients cannot perform surgical operations. Conventional external radiotherapy is limited by the tolerable dose of normal human tissues and spinal cord, and the treatment dose cannot be further increased, and it is difficult to reach the lethal dose of tumors, and tumors are prone to recurrence.

Intermediate bone tumors and benign bone tumors of the spine are usually younger and more common in adolescents. Clinically, local symptoms are mild and the changes are not obvious. Usually, there are no systemic symptoms and the course of the disease is often longer. Most primary malignant bone tumors of the spine have an older age and are more common in adults, the local symptoms are severe and progressively worse, and there may be systemic symptoms. The course of the disease changes significantly in a short period of time, but the age of onset of lymphoma is relatively young. Spinal metastatic tumors account for about 50% of spine bone tumors. They are the most common malignant bone tumors of the spine. The clinical and imaging findings are typical, and the diagnosis is not difficult. There are many types of primary spine bone tumors, and they are relatively rare. Moreover, most clinical and imaging studies lack characteristic changes, and diagnosis is often difficult. In recent years, domestic and foreign scholars have conducted various imaging studies, but the number of cases is often small. So far, the research on imaging diagnosis of spine bone tumors has not been in-depth, and there are not many studies on the imaging signs of primary spine bone tumors.

This article mainly focuses on the retrospective analysis of the plain film, CT, and MRI manifestations of cases of spinal bone tumors. Moreover, this article further summarizes the imaging characteristics of spine bone tumors, improves the imaging diagnosis level of spine bone tumors, and subdivides each pathological type for independent diagnosis and treatment analysis. This study hopes to analyze the clinical and imaging manifestations of different pathological types based on the new classification of bone tumors through a larger group of cases, so as to provide a new reference for daily imaging diagnosis. Spinal bone tumors can be divided into different histopathological types according to the dominant cellular components in tumor tissues, including metastatic bone tumors, plasma cell myeloma, primary non-Hodgkin's lymphoma, and giant cell tumor of bone. Among the many pathological types, metastatic bone tumors account for the vast majority. Therefore, clinical manifestations and imaging diagnosis mostly focus on the characteristics of malignant bone tumors. The incidence of males is higher than that of females, and most of them occur in the thoracic and lumbar spine. It is combined with the imaging technology to analyze the pathology of spine bone tumors, and provided a theoretical reference for the clinical diagnosis and treatment of spine bone tumors.

## 2. Related Work

As the incidence of vertebral tumors increases year by year, its treatment has gradually attracted people's attention. Spinal tumors are divided into primary tumors and secondary tumors according to their sources. Among them, secondary is more common than primary, and hemangioma, myeloma, giant cell tumor of bone, etc. are the more common primary tumors [5]. Secondary tumors are mostly metastatic tumors. It has been reported in the literature that the spine has become the most common site for bone metastases due to its abundant blood supply, accounting for about 50% of the body's bone metastases. The spine has a special anatomical structure and is adjacent to important organs and large blood vessels in the abdominal cavity. The spinal canal contains the spinal cord and there are nerves on both sides. Therefore, complete removal of the diseased vertebral body will reduce the stability of the spine. Moreover, open surgery for spinal vertebral body tumors is more difficult and riskier, and it has always been a difficult point in the treatment of spinal tumors [6].

At present, nearly 8% of benign bone tumors are located in the spine or sacrum. The age of onset is more common in adolescents, and 60% of spine tumors occur in 20-30 years old. The most common complaints are pain, localization, or radiating pain. Osteoid osteoma and osteoblastoma often have nocturnal pain, and salicylic acid can be used as an analgesic, which is one of its characteristics [7]. Back pain is rare in children, and this main complaint should be paid attention to. It is generally believed that the possibility of benign tumors should be paid attention to for pain after minor trauma. Intervertebral disc herniation in children and adolescents is also rare. If there is radicular pain, the possibility of tumor should also be ruled out [8]. According to observations, 37% of benign cervical spine tumors have root pain. Among the signs of benign spinal tumors, local tenderness is not specific. We need to pay attention to the following characteristics of scoliosis: rapid development of scoliosis with pain; stiffness of the spine; more uncompensated balance curvatures above and below the curvature of the lesion; no vertebral body rotation and wedge change on X-rays. These are different from idiopathic scoliosis. About one-third of the tumors that occur in the cervical spine have torticollis. When a tumor is compressed or a pathological fracture occurs, which affects the nerve structure, it produces signs of the nervous system, such as radicular pain and signs of impaired nerve function. Moreover, it can produce myelopathy manifestations of impaired spinal cord function, such as changes in sensation, movement, reflex, and pyramidal tract signs. In particular, tumors in the cervical and thoracic vertebrae are likely to cause damage to the function of the spinal cord. Lumps in the spine are most easily found in the cervical and sacral spine, and are easier to touch than lumps in the thoracic and lumbar spine. Therefore, careful palpation and oropharyngeal examination are required, and anal examination should also be performed [9].

Primary malignant bone tumors of the spine are rare. However, 80% of adult spinal tumors are malignant tumors. The main clinical manifestation is pain, and nocturnal pain is a common complaint. Pain is sometimes related to activity, but when the tumor causes pathological fractures, the pain has nothing to do with activity, and rest does not relieve [10]. When the nerve root is affected, persistent back pain and radicular pain occur. One-fifth of cervical and lumbar tumors have unilateral radicular pain, while thoracic spine tumors are likely to cause compression of the spinal cord or bilateral radicular pain. The main signs are caused by tumor compression of the spinal cord or nerve roots [11]. According to the different parts of the spine, the nervous system has different manifestations. If the spinal cord is compressed, there will be corresponding signs of upper motor neuron damage. If the lesion is below the cauda equina, there will be signs of lower motor neuron damage [12]. Although these signs are not specific, they are meaningful for judging the location of nerve damage. Malignant primary spinal tumors can also have systemic symptoms, such as myeloma, lymphoma, and Ewing's sarcoma, and may have weight loss, low-grade fever, general fatigue, etc., and cachexia may occur in the late stage. Local lumps can also be seen. For example, cervical chordoma can be found in pharyngeal masses, and sacrococcygeal chordoma can be found in anal examination [13]. Primary benign tumors of the spine mostly occur in a single vertebral body, of which the thoracic spine is the most common, followed by the sacral spine and lumbar spine, and the cervical spine is relatively rare. On the TWI image, it shows uniform or uneven low signal, and the damage margin is clear, accompanied by reactive osteogenesis. Generally, the cortical bone is intact or the bone shell is formed after compression damage. The tumor does not damage the intervertebral disc, and most of them show uniform enhancement. There are also few paravertebral soft tissue masses, and a few tumors can show masses, ossification, or involve adjacent vertebrae. Primary benign tumors of the spine have their own characteristics due to their different natures [14].

Vertebral hemangioma generally has typical X-ray manifestations, and the vertebral body changes in a fence shape. This is due to the absorption of the transverse trabecular bone, the remaining longitudinal trabecular bone being pushed by the expanded blood vessels and the compensatory thickening due to weight bearing. Some hemangioma showed grid-like changes, and MRI showed high signal with dots and low signal, and the enhanced scan was significantly enhanced. Aneurysmal bone cysts are cystic swelling changes, and the lesions can be single or multilocular structures with clear boundaries, and they have or without bony septal or bone crest [15]. Significantly swollen lesions often break through the cortical bone and grow into soft tissues to form soft tissue masses. Moreover, some aneurysmal bone cysts can often see characteristic fluid levels in cystic lesions [16]. The liquid-liquid level that appears on CT and MRI is a more characteristic change of aneurysmal bone cyst. However, it is not unique to aneurysmal bone cysts, and lesions with bleeding in the lesion and separation of blood cells and plasma can produce this sign [17].

## 3. Methods and Information

There are 25 cases in this group, and a total of 30 vertebral bodies, including 12 males and 13 females. The age range is 38-81 years old, and the average age is 63.5 years old. The patient's clinical symptoms include varying degrees of pain, percussive pain, and movement disorders in the vertebral body. The lesions include 2 lumbar 5 vertebrae, 3 lumbar 4 vertebrae, 3 lumbar 2 vertebral bodies, 5 lumbar 1 vertebral body, 5 thoracic 12 vertebral bodies, 3 thoracic 11 vertebral bodies, 3 thoracic 10 vertebral bodies, and 1 thoracic 9 vertebral bodies. The etiology is as follows: 3 cases of myeloma, 5 cases of hemangioma, 1 case of aneurysmal bone cyst, 15 cases of metastasis. The primary source of thoracolumbar metastases: 4 cases of breast cancer, 4 cases of lung cancer, 4 cases of gastric cancer, 3 cases of prostate cancer. X-ray examinations are performed before the operation, CT and MRI examinations are performed on the diseased vertebral body, and some patients with conditional vertebral body metastases require ECT examination.

### 3.1. Inclusion Criteria

Patients without severe hemorrhagic, coagulative disease or severe lung disease, with stable vital signs, and physical conditions that can tolerate surgery; patients with varying degrees of vertebral collapse and bone destruction in the diseased vertebrae shown by ordinary plain films; patients with osteolytic destruction of the diseased vertebrae shown by CT and MRI; patients with malignant tumors undergoing radiotherapy before surgery.

### 3.2. Exclusion Criteria

Terminal patients with extreme weakness in the advanced stage of cachexia; patients with spinal cord infringement and obvious spinal cord and nerve root damage on MRI; patients with severe cardiopulmonary dysfunction and other patients who cannot tolerate surgery; patients who cannot tolerate surgery such as severe cardiopulmonary dysfunction; patients who have symptoms of infection in the operating area or the whole body; and patients who cannot cooperate with surgery due to mental disorders. It used a special PVP needle with a beveled puncture surface for puncture, and a matching PVP syringe for bone cement injection. Intraoperative monitoring equipment uses a large-scale digital subtraction angiography (DSA). The bone cement material is polymethyl methacrylate (PMMA), which comes from Tianjin Institute of Synthetic Materials Industry. It is necessary to inform the patients that they need to do prone position exercises for a long time before the operation, so that the patient's cardiopulmonary function can adapt to the intraoperative position. Another advantage is that the prone position can be used to make the partially compressed vertebral body repositionable. During the operation, the prone position was adopted, lidocaine was used for local infiltration anesthesia, and it was performed under the supervision of a large digital subtraction angiography (DSA). The puncture needle should generally be located 2-3 cm next to the spinous process, the outer edge of the pedicle projection. In addition, the puncture needle and the sagittal plane of the vertebral body form an angle of about 15-20 degrees, and gradually enter the vertebral body along the pedicle, and enter and perform fluoroscopy. The bone cement is prepared under vacuum conditions. When the bone cement has solidified to a viscous stage, the prepared bone cement is slowly injected into the vertebral body with a special injection device under DSA monitoring. 4-6 ml PMMA bone cement was injected into the diseased vertebrae with intact posterior edge of the vertebral body, and <3 ml PMMA bone cement was injected into the diseased vertebrae with relatively incomplete posterior edge of the vertebral body. It is necessary to observe while injecting. Once the bone cement leaks to the surrounding area, the operation should be terminated immediately. A total of 28 vertebrae are treated, and ECG monitoring is applied during the operation. After the operation, the patient was supine on the pillow for 4-6 hours. After 2-3 days, the patient can properly perform functional exercises under the protection of the thoracic, waist, and back brace, and review the injection and distribution of bone cement 3 days after surgery. Antibiotics should be used for 3 days to prevent infection, and regular anti-tumor radiotherapy or chemotherapy should be given at the same time.

### 3.3. Standard Radiotherapy

The indication of traditional radiotherapy is painful spinal metastases without mechanical instability and nerve damage. The total dose of radiotherapy is 25-40Gy, which is completed in 8-20 days. Its role is to relieve the pain of metastatic tumor lesions, prevent vertebral body collapse and pathological fractures, and delay the damage of nerve function. The effect of radiotherapy depends on the total dose of radiation and the sensitivity of the tumor to radiotherapy. For solitary metastatic carcinoma with obvious mechanical instability, radiotherapy alone is not sufficient. Radiation therapy can cause nerve damage in patients with recurrence of spinal metastases, especially the possibility of myelitis, so patients with recurrence of spinal metastases cannot receive radiotherapy again. The accuracy of traditional radiotherapy is limited, and the tolerance of the spinal cord is low. The total dose that can tolerate radiotherapy is lower than the optimal total dose of radiotherapy. Some scholars have proposed whether it is possible to change fractional low-dose radiotherapy to single high-dose radiotherapy. However, the meta-analysis found that fractional radiotherapy with a total dose of 8-10 Gy and single radiotherapy have the same analgesic effect and patient survival time, and many single radiotherapy patients need to be treated again.

This article uses image analysis to analyze spine tumors, as shown in Figures 1–4.

Through the evaluation of the quality of life, it is found that the quality of life of patients before and after the treatment of percutaneous vertebroplasty has significant changes. After the treatment, the physical state, mental state, and quality of life have been significantly improved, as shown in Table 1.

After treatment by percutaneous vertebroplasty, no displacement of the treated vertebrae has been found, that is, the original physiological curvature changes, angulation, and spondylolisthesis have not been aggravated. Moreover, there were no symptoms of further collapse of the treated vertebral body, kyphosis, compression of the spinal cord or nerve roots, or paralysis.

## 4. Analysis and Discussion

The treatment of spinal tumors has always been a difficult clinical problem. The unbearable and unhealed pain and vertebral fractures caused by tumor invasion have severely reduced the quality of life of patients. Whether or not to operate and what kind of surgical procedure to adopt has always been a question of concern to scholars. In recent years, with the continuous development of spinal surgery technology and the increasing renewal of tumor treatment concepts, more and more patients with spinal tumors have begun to receive surgical treatment. Due to the shortcomings of large trauma, many complications, and long postoperative recovery period, open surgery is not suitable for the treatment of spinal tumors, especially the treatment of multiple spinal metastases.

PVP, as a relatively safe and effective spine minimally invasive surgery technique, can quickly relieve pain, with small surgical trauma and simple operation. Moreover, it can usually be completed under local anesthesia, and only need to stay in bed for a few hours after surgery to get out of bed. It is widely used in clinical practice, even as the first choice for the treatment of spinal tumors, and has achieved good results. There are several widely recognized theories regarding the analgesic principles of PVP at home and abroad [18]: ① bone cement polymethyl methacrylate (PMMA) is a new type of polymer material. The high heat generated when the monomer polymerizes can damage the local sensory nerve endings; ② the chemical properties of bone cement itself can also destroy the damage of local sensory nerve endings; ③ polymethylmethacrylate (PMMA) itself can kill tumor cells and reduce the damage to bone tissue caused by stimulating factors released by tumors; ④ the pressure reduction in the lesion after puncture is related; ⑤ bone cement (PMMA) has the effect of inhibiting tumor growth; ⑥ bone cement (PMMA) monomer is toxic and can directly kill tumor cells. After the preoperative radiotherapy of patients with spinal tumors, the formation of adhesion bands and the proliferation of fibrous tissue in the local defect area of the diseased vertebra were observed during open surgery. In patients with spinal metastases, local radiotherapy to the operation area before percutaneous vertebroplasty can cause fibrosis of the diseased vertebral tumor tissue. In the diseased vertebral body, especially in the case where the posterior edge of the vertebral body is destroyed and infiltrated by tumor tissue in a large area, the hyperplastic fibrous tissue can prevent the leakage of uncured bone cement into the spinal canal to a certain extent, thereby reducing the risk of surgery and reducing the occurrence of postoperative complications. This is the guarantee that there is no case of bone cement leaking into the spinal canal in this group of operations. For patients with simple osteoporotic fractures and large-scale bone defects on the posterior edge of the diseased vertebra, percutaneous vertebroplasty and bone cement injection are not recommended. In order to improve the strength of the vertebral body after a simple fracture, the dose of bone cement cannot be reduced. At this time, the spinal canal and the vertebral body are directly connected, which greatly increases the risk of bone cement leakage. Precautions during surgery: relevant literature has reported [19] PVP surgery may cause complications of pulmonary embolism and bone cement leakage. Strictly controlled bone cement injection timing can avoid the occurrence of this symptom. From the beginning of the preparation of the bone cement to the complete solidification of the bone cement, there are roughly three intervals: ① the thinning period: it is approximately within 1 minute after mixing and mixing. During this period, bone cement still has relatively large fluidity. Injecting the vertebral body at this stage, if we are not careful, it is easy to cause leakage of bone cement. ② Viscous period: it refers to within 1 minute to 3 minutes after mixing and blending. This is the best time for bone cement injection. Beyond this period, the viscosity of the bone cement increases and the bolus injection becomes difficult, and even the operation fails due to the inability to boluse the injection. ③ Setting and hardening period: this period is very important and is the key stage for bone cement to produce therapeutic effects. The increase in the strength of bone cement and the generation of heat generation are formed at this stage.

There are two commonly used PVP puncture needle tips [20], including rhombus and oblique surface. When a diamond-shaped needle is used to inject bone cement into the vertebral body, it diffuses around, and when a beveled needle is used to inject bone cement into the vertebral body, it can selectively diffuse to one side. According to our clinical experience, patients with spinal metastases with large-area defects on the posterior edge of the vertebral body at the lesion should choose a puncture needle with a beveled needle for injection. If the inclined surface faces the defect, the chance of bone cement leakage will increase; otherwise, the chance of leakage will be small. By rotating the angle of the needle to inject the bone cement in the opposite direction of the vertebral body defect not only can the success rate of the operation be improved, but also the safety of the operation can be greatly improved. When injecting bone cement, you need to apply pressure slowly to avoid injecting the bone cement during the thinning period and reduce the risk of bone cement leakage. At the same time, real-time imaging monitoring is performed. Once bone cement leakage occurs, the operation should be terminated immediately. The relationship between the dose of bone cement injection and clinical efficacy: there have been many reports in the literature on the dose of bone cement injected into the target vertebral body. Too little injection volume will not achieve satisfactory clinical results, and too much injection volume will greatly increase the incidence of complications. The literature [21] concluded through clinical trials that the filling amount of bone cement reached 14% of the entire vertebral body volume to restore the vertebral body stiffness to the ideal state. Moreover, too large a dose of bone cement cannot achieve the best biomechanical effect on the diseased vertebra. In the actual clinical treatment process, we found that the amount of bone cement injected is not directly proportional to the clinical analgesic effect. Moreover, it is proportional to the probability of bone cement leakage and the strength of the vertebral body. For patients with simple osteoporotic compression fractures, not only should the pain be relieved, but also the hardness and strength of the diseased vertebrae should be restored. Therefore, the dosage of bone cement should be increased as much as possible. For patients with vertebral tumors, while pursuing analgesic effects, more attention should be paid to reducing the occurrence of complications. Relevant literature has reported that blindly pursuing analgesic effect and ignoring the occurrence of complications and blindly increasing the injection dose of bone cement are very undesirable. Excessive bone cement injection will greatly increase the incidence of re-fractures of adjacent vertebral bodies after surgery. In order to reduce bone cement leakage, different surgical methods and bone cement materials have been widely compared. When the cement viscosity is different, its flow stability is different, and the flow stability of high-viscosity bone cement is better. In the literature [22], 14 diseased vertebrae of 9 patients with thoracolumbar vertebral metastases are treated by percutaneous small-dose bone cement infusion. The average injection volume of each vertebral body is 4.8 ml, the postoperative pain is relieved immediately, and there is no case of bone cement leakage. The above is the theoretical basis for this group of patients with spinal tumors to undergo percutaneous bone cement injection to reduce local pain and improve the quality of life. The postoperative weight-bearing of the vertebral body needs to be supported by long-term wearing of thoracic, lumbar, and back braces. We have reason to believe that for patients with intact vertebral posterior spine tumors, the amount of bone cement injection should be 4-6 ml, and for patients with incomplete posterior edges, the amount of bone cement injection should be less than 3 ml. This dose has been able to achieve clinically satisfactory results. Simply increasing the amount of bone cement injected will not further relieve the pain, especially for patients with defects on the posterior edge of the vertebral body; it will greatly increase the risk of bone cement leakage. In literatures [23] and [24], there are studies on preoperative radiotherapy and postoperative stent wearing. It is reported in the literature that in the cases of spinal tumors treated by percutaneous vertebroplasty, some patients developed adjacent vertebral fractures after the filled bone cement leaked into the surrounding tissue. We believe that this occurrence is not only related to the aggravation of tumor invasion, but may also be related to the lack of regular radiotherapy before surgery and effective brace protection after surgery. In particular, during preoperative radiotherapy, effective radiotherapy can damage diseased tissues (and involve normal tissues at the same time). In open surgery for patients with spinal metastases after preoperative radiotherapy, it was found that there was fibrous tissue hyperplasia and adhesion formation in the defect area. Compared with simple osteoporotic fractures with large-scale bone defects on the posterior edge of the vertebral body, radiotherapy at the preoperative area of PVP can cause fibrosis of the tumor tissue of the diseased vertebral body. After a large area of bone in the posterior edge of the diseased vertebral body is destroyed and moisturized by the tumor tissue, the locally proliferated fibrous tissue can prevent the unsolidified bone cement from entering the spinal canal to a certain extent, thereby reducing the risk of surgery. Wearing a brace after surgery can play a supporting role. This supporting role can not only effectively relieve the pressure on the spine and its surrounding soft tissues during daily activities. Moreover, to some extent, it can promote the regeneration of normal tissues.

## 5. Summary

We have reason to believe that radiotherapy to local tissues before percutaneous vertebroplasty and wearing a brace to support the weight and share the pressure are important guarantees for good results in this group of cases. The purpose of surgery for patients with spinal tumors is to remove the lesion to the greatest extent, maintain the stability of the spine, restore nerve function as much as possible, prevent spinal cord injury, relieve pain, improve the quality of life of patients, and prolong survival. At present, open surgery alone is not the first choice for the treatment of spinal tumors. For patients with spinal metastases and giant cell tumors of bone, because of their high recurrence rate, simply scraping the lesions will not solve the actual problems. Although large-area resection of the tumor can reduce the local recurrence rate, the patient's own mobility is significantly impaired, and the stability is not as good as before the operation. Moreover, domestic and foreign experts on the reconstruction and repair of spinal stability after total spine lumpectomy are further exploring and researching. Literature [25] proved that long-segment fixation or anterior and posterior fixation can provide better stability through biomechanical experiments. However, this operation is more expensive than percutaneous vertebroplasty, and the trauma is relatively large. It is especially not suitable for the elderly and frail patients. At present, the evaluation of the efficacy of percutaneous vertebroplasty in the treatment of vertebral body tumors is mainly based on the degree of pain relief, but the evaluation of clinical treatment effects through pain relief alone cannot truthfully and fully reflect the overall quality of life of patients.

## 6. Conclusion

This article analyzes the clinical diagnosis and treatment of spinal bone tumors based on imaging. Moreover, this study developed a health status questionnaire and adopted a scoring method for comprehensive assessment. The purpose is to show that by combining preoperative radiotherapy and postoperative bracing, bone cement injection to treat vertebral tumors, especially small doses of bone cement injected into patients with spinal tumors with defects on the posterior edge of the vertebral body, can immediately obtain satisfactory pain relief. Moreover, it has an inhibitory effect on local tumors to a certain extent, which greatly improves the quality of life of patients. Although there is new bone formation at the posterior edge of the vertebral body in this group of cases of spinal metastasis, whether small doses of PVP can promote new bone formation needs further research to confirm. This article believes that early and aggressive treatment of spinal metastases with large-scale defects in the posterior edge should be taken. In other words, regular radiotherapy, low-dose bone cement PVP surgery, and postoperative brace protection are required before surgery.

## Figures and Tables

**Figure 1:** Case 1.

**Figure 2:** Case 2.

**Figure 3:** Case 3.

**Figure 4:** Case 4.

**Table 1:** Quality of life score results before and after treatment.

	Physical state	Mental state	Overall quality of life
Before PVP	85.4 ± 64.5	93.5 ± 63.9	178.9 ± 128.4
After PVP	159.1 ± 59.3	186.1 ± 85.2	345.2 ± 134.5
*T* value	1.34	1.81	1.66
*P* value	0.009	0.014	0.002

## Data Availability

The data used to support the findings of this study are included within the article.
